# Changes and Influencing Factors of Cognitive Impairment in Patients with Breast Cancer

This article has been retracted.

**DOI:** 10.1155/2021/7278853

**Published:** 2021-10-28

**Authors:** Huixia Cui, Xusheng Shi, Xiaoxiu Song, Wenlu Zhang

**Affiliations:** ^1^College of Nursing, Jinzhou Medical University, Jinzhou, Liaoning 121001, China; ^2^Department of Intensive Care Medicine, Liaocheng People's Hospital, Liaocheng, Shandong 252000, China; ^3^Department of Radiation Oncology, The First Affiliated Hospital of Jinzhou Medical University, Jinzhou, Liaoning 121001, China

## Abstract

**Objective:**

To investigate the changes in cognitive function and its influencing factors in patients with breast cancer after chemotherapy, to provide a scientific basis for further cognitive correction therapy.

**Methods:**

In this study, general information on age, marital status, and chemotherapy regimen was collected from 172 breast cancer chemotherapy patients. 172 patients with breast cancer undergoing chemotherapy were investigated by convenience sampling method, and the subjects were tested one-on-one using the Chinese version of the MATRICS Consensus Cognitive Battery (MCCB) computer system.

**Results:**

The mean value of standardized t-value of cognitive function and its abnormal dimensions in breast cancer patients undergoing chemotherapy were MCCB total cognition (66.3%, 36.99 ± 13.06, abnormal), working memory (73.3%, 36.84 ± 10.25), attention and alertness (70.3%, 37.20 ± 12.50), social cognition (65.1%, 39.54 ± 10.17), and visual memory (61.6%, 42.19 ± 9.38). A comparison of cognitive function among breast cancer chemotherapy patients with different demographic characteristics showed that differences in place of residence, educational level, monthly income, timing of chemotherapy, chemotherapy regimen, and chemotherapy times may be associated with abnormal cognitive function. Further multiple linear regression analysis was performed and the results showed that there was a linear regression between literacy, number of chemotherapy sessions, monthly personal income, and cognitive function.

**Conclusion:**

Cognitive impairment is common in patients with breast cancer after chemotherapy. Nurses should pay attention to the cognitive function changes and intervention of patients with breast cancer after chemotherapy, to prevent the changes of cognitive function and promote the rehabilitation of patients.

## 1. Introduction

Breast cancer is already the most common malignant tumor in women with the highest incidence [1]. In 2018, it is estimated that there are about 2.1 million new cases of breast cancer worldwide, accounting for 25% of all new cases of malignant tumors [2]. In recent years, the incidence and mortality of female breast cancer in China has increased year by year, and the disease burden of breast cancer patients has also increased year by year. At present, surgery combined with postoperative chemotherapy is still the first choice for the treatment of breast cancer, but chemotherapy drugs are used in the treatment of diseases. At the same time, there are many adverse reactions, which brings great pain to patients [3]. Studies have shown that chemotherapy will cause not only leukocytosis, nausea, vomiting, loss of appetite, bone marrow suppression, hair loss, and so on, but also severe cognitive decline [4]. Chemotherapy-related cognitive impairment [5] (chemotherapy-related cognitive impairment, CRCI), also known as chemotherapy brain (chemobrain) or chemotherapy fog (chemofog), is refered to the memory of patients with malignant tumors during or after chemotherapy and the decline of cognitive functions such as power, executive ability, language ability, reasoning ability, and visual space ability [6]. The pathogenesis of CRCI is not yet clear. Studies have confirmed that it is related to a variety of factors, including changes in estrogen levels, inflammation, and DNA factors.

The occurrence of CRCI not only affects the frequency of social interaction and the efficiency of work for breast cancer patients but also has a serious impact on the patient's ability to perform daily activities, which can be physically and mentally devastating and have a negative impact on family harmony. Currently, most of the studies on cognitive impairment in China focus on elderly patients, stroke patients, and other populations, and there are fewer studies on cognitive impairment and its influencing factors in breast cancer chemotherapy patients [7]. This study, therefore, investigates breast cancer chemotherapy patients, using a neuropsychological test as a research tool and a computerized measurement platform to enable the implementation of computer-assisted data for brain function tests and the implementation of validated cognitive function sets for patients in hospitals. This is to provide a clearer understanding of the current status of CRCI in breast cancer chemotherapy patients and to analyze its influencing factors, to provide a scientific basis for further cognitive remediation treatment.

## 2. Objects and Methods

### 2.1. Object

Convenience sampling was used to investigate the subjects who met the inclusion criteria in the First and Third Affiliated Hospitals of Jinzhou Medical University from October 2018 to March 2020. Inclusion criteria: (1) patients with histopathologically diagnosed breast cancer and undergoing chemotherapy; (2) no hearing, vision, language, and other dysfunctions and having certain expression and reading ability; and (3) voluntarily participating in the research of this subject. Exclusion criteria: (1) patients with advanced cachexia; (2) patients with cognitive impairment prior to receiving chemotherapy treatment; (3) patients with obvious anxiety, depression, and other mental illnesses; (4) patients taking drugs related to cognitive function; (5) patients with intracranial abnormalities and intracranial metastases on MRI or CT examination of the head; (6) combined with severe heart, liver, kidney, brain, and hematopoietic system diseases. 206 breast cancer chemotherapy patients participated in this study, of whom 34 did not complete this study, for a final sample size of 172. The general information is shown in Table 1.

### 2.2. Method

#### 2.2.1. Survey Tools

1. The general information survey form was designed by the research themselves according to a large amount of literature, mainly including age, marital status, education level, personal monthly income, surgical method, disease stage, chemotherapy regimen, chemotherapy cycle, etc. 2. The Chinese version of the computer system for MATRICS Consensus Cognitive Battery (MCCB) was introduced from the United States in 2009 by Beijing Huilongguan Hospital. After translation and back translation, the Chinese version of MCCB was revised and completed. Later, Beijing Huilongguan Hospital organized experts to conduct tests, standardization, and computerization. In all MCCB subtests, except for the visual memory test, which is subjectively scored by the rater, other subtests are automatically scored by computer programs. As long as the main tester operates according to the regulations, there is no need for the main tester to score by time. The MCCB is an individual cognitive function test, which requires one-to-one testing between the examiner and the subject. The examiner needs to have certain qualifications and undergo a rigorous training before the evaluation. According to the results of the cognitive function test, the number of standard deviations compared with the norm is used to determine the degree of cognitive deficits.

#### 2.2.2. Survey Method

This study was reviewed and approved by the Ethics Committee of Jinzhou Medical University. Convenience sampling was used to investigate the subjects who met the inclusion criteria in the First and Third Affiliated Hospitals of Jinzhou Medical University from October 2018 to March 2020 and solicited the test subjects. After the participants and their family members agree, the researchers explained the test procedures and requirements in detail to the subjects and conducted one-to-one computer system tests on the subjects.

#### 2.2.3. Statistical Methods

The data was checked by two persons and entered into SPSS 21.0, and statistical analysis was carried out. The statistical data were expressed as rates and composition ratios (*n*, %) using the chi-square test, while the measurement data were expressed as mean ± standard deviation (mean ± SD), using *t*-test between two groups and one-way variance (F) test between multiple groups. Pearson's model was used for correlation analysis and the multiple linear regression model for multifactor analysis; *P* < 0.05 was considered statistically significant.

## 3. Results

### 3.1. Analysis of the Current Status of Various Dimensions and Subtest Results of Cognitive Function in Patients with Breast Cancer Chemotherapy

#### 3.1.1. Analysis of the Current Status of Various Dimensions of Cognitive Function in Patients with Breast Cancer Chemotherapy

The processing speed score of breast cancer chemotherapy patients is (48.83 ± 10.73), the working memory score is (36.84 ± 10.25), and the speech learning score is (44.67 ± 10.90) as shown in Table 2.

#### 3.1.2. Ratio Analysis of the Current Status of Various Dimensions and Subtest Results of Cognitive Function in Patients with Breast Cancer

Chemotherapy among the 172 breast cancer patients undergoing chemotherapy: the percentages of cognitive impairment in various dimensions, from high to low, were working memory (73.3%), attention/alertness (70.3%), social cognition (65.1%), and visual memory (61.6%), verbal memory (34.3%), processing speed (27.3%), reasoning and problem-solving ability (23.3%), and MCCB cognitive total score (66.3%), as shown in Table 3.

### 3.2. Comparison of Cognitive Function of Breast Cancer Patients Undergoing Chemotherapy with Different Demographic Characteristics

The results of the comparison of cognitive function in breast cancer chemotherapy patients with different demographic characteristics showed that differences in place of residence, literacy, monthly income, timing of chemotherapy, chemotherapy regimen, and chemotherapy times may be associated with abnormal cognitive function (*p* < 0.05). See Table 4 for details.

### 3.3. Multiple Linear Regression Analysis of Cognitive Function in Patients with Breast Cancer Chemotherapy

The MCCB score of patients with breast cancer chemotherapy was used as the dependent variable, and the statistically significant variables in the univariate analysis were used as independent variables to perform multiple linear stepwise regression analysis (*α*in = 0.05, *α*out = 0.10). The analysis revealed that education level, chemotherapy times, and personal monthly income (see Table 5 for assignments) were risk factors for cognitive function in breast cancer chemotherapy patients (*p* < 0.05), as shown in Table 6.

## 4. Discussion

### 4.1. Analysis of the Status Quo of Cognitive Function in Breast Cancer Patients Undergoing Chemotherapy

Tables 2 and 3 of the results of this study show that the total standardized T score of MCCB for cognitive function in breast cancer patients is 10 to 63 points, and the average T score is 36.99 ± 13.06. The result is abnormal, and the cognitive function of breast cancer patients undergoing chemotherapy is impaired. It shows that the cognitive function of breast cancer patients undergoing chemotherapy is generally impaired, which is basically consistent with previous studies. Huang's [8] study showed that 19% to 78% of breast cancer chemotherapy patients experienced varying degrees of decline in cognitive function. Most studies [9] have shown that the cognitive function of breast cancer patients undergoing chemotherapy is impaired, which has attracted the attention of clinical medical staff. In clinical practice, medical staff should pay attention to the cognitive status of patients, analyze its influencing factors, and conduct cognitive interventions for patients to improve the quality of life of patients.

### 4.2. Influencing Factors of Cognitive Function Changes in Breast Cancer Patients Undergoing Chemotherapy

#### 4.2.1. Cognitive Function Analysis of Breast Cancer Chemotherapy Patients with Different Education Levels

In this study, patients with different educational levels (*F* = 73.322, *p* < 0.001), elementary school, junior high school, high school, and university degrees had standardized T scores of 25.50 ± 9.37, 29.12 ± 8.95, 47.09 ± 7.60, and 47.77 ± 12.10, respectively, indicating that the higher the educational level, the better the cognitive function. This is consistent with the results of other scholars on the cognitive function and education level of breast cancer chemotherapy patients [10]. The results of this study show that there are significant differences in cognitive function among patients with different education levels. Patients with higher education levels have better cognitive functions. The possible reason is that patients with higher educational levels can better communicate with medical staff, strive for more social support, and reduce their negative emotions. Patients with a low level of education have more conservative thinking, less communication with others, and greater psychological pressure. This requires medical staff in clinical practice to give corresponding cognitive psychological interventions according to the education level of the patients and to provide the patients with the best quality care.

#### 4.2.2. Analysis of the Relationship between Different Monthly Income and Cognitive Function

Personal monthly income (*F* = 9.085, *p* < 0.001): the average standardized T-scores of cognitive function of patients from low to high personal monthly income groups were (32.47 ± 8.44), (30.61 ± 12.27), (41.32 ± 13.87), and (41.50 ± 11.34), indicating that the higher the monthly income, the better the cognitive function. At the same time, the level of education and personal monthly income are synergistically related. Generally, the higher the level of education means the higher the monthly income. Patients living in cities have better cognitive functions than those living in rural areas. The possible reason is that patients living in cities have more convenient access to disease information, can participate in more social activities, relieve their negative emotions, and further improve their cognitive function.

#### 4.2.3. Analysis of the Relationship between Chemotherapy (Timing of Chemotherapy, Chemotherapy Regimen, Chemotherapy Times) and Cognitive Function of Breast Cancer Patients

The results of this study showed that the average cognitive standardized T scores of patients undergoing preoperative and postoperative chemotherapy were 33.89 ± 13.14 and 38.76 ± 13.68, respectively, indicating that the cognitive function of patients undergoing preoperative chemotherapy was worse than that of patients undergoing postoperative chemotherapy (*t* = −2.205, *p* = 0.029); patients with TP (paclitaxel, cisplatin) chemotherapy regimens have the lowest average cognitive standardized T score, and the average value is 29.48 ± 14.45, which is worse than patients with other chemotherapy regimens (*t* = 2.945, *p* = 0.035). The more the chemotherapy times, the worse the cognitive function (*t* = 23.659, *p* < 0.001). One scholar [11] studied the effect of three different chemotherapy regimens on the cognitive function of breast cancer patients, and the results showed that the EC-T regimen (epirubicin+cyclophosphamide sequential docetaxel) is more likely to cause cognitive impairment in patients than the FEC regimen (epirubicin, fluorouracil, cyclophosphamide) and the TC regimen (docetaxel, cyclophosphamide). Chemotherapy is the most important risk factor for cognitive dysfunction in breast cancer patients. Chemotherapy for breast cancer patients, including timing of chemotherapy, chemotherapy regimen, and chemotherapy times, will have an important impact on the cognitive function of breast cancer patients undergoing chemotherapy [12]. However, some studies [13] have shown during the 0–3 chemotherapy cycles, the patient's cognitive ability gradually declines but some improve in cognitive ability during cycles 4–7 and above. The possible reason for the difference in results is related to the different measurement tools and sample size in this study, and future studies should be conducted with larger samples to further check the research hypothesis.

#### 4.2.4. Analysis of the Relationship between Cancer Factors (Pathological Type, Cancer Stage) and Cognitive Function

The results of this study showed that the average standardized T-score of cognitive function of patients with carcinoma in situ (39.55 ± 16.76) was higher than that of patients with invasive cancer (36.93 ± 13.52) and metastatic cancer (36.73 ± 11.99), indicating that the cognition function of patients with mild pathological types is better. According to different clinical stages, the average cognitive function T scores from high to low are stage I (40.12 ± 17.61), stage II (39.16 ± 13.75), stage III (36.48 ± 11.29), and stage IV (32.94 ± 12.26), indicating the condition of the disease was lighter, the function was better. At present, most research is carried out after patients undergoing chemotherapy or surgery. A few scholars pay attention to the cognitive function of patients before treatment. Studies abroad [14] found that patients have symptoms of cognitive decline before surgery. And the incidence rate is as high as 40%. Chemotherapy-related cognitive dysfunction has different manifestations in different patients, pathological types, and cancer stages and can appear at different stages of cancer treatment. Studies by scholars have also shown that the percentages of cognitive impairment in breast cancer patients before, during, and after chemotherapy are 40%, 75%, and 60%, respectively. Therefore, breast cancer itself can also affect the cognitive status of breast cancer patients. Clinical medical staff can take different cognitive correction nursing measures according to the patient's different pathological types, different clinical stages, and whether they have metastasis and should take more targeted prevention and treatment of cognitive dysfunction in breast cancer patients undergoing chemotherapy.

#### 4.2.5. Analysis of the Relationship between the Treatment of Breast Cancer Patients (whether Surgery, Operation Method) and Cognitive Function

The results of this study showed that the average T-scores of breast cancer patients who underwent surgery and those who did not undergo surgery were (36.86 ± 13.27) and (39.07 ± 15.76), respectively, indicating that the cognitive function of patients who underwent surgery was worse than that of patients who did not undergo surgery. From the point of view of the standardized T-score of cognitive function, the cognitive function of patients with breast-conserving surgery (39.67 ± 12.00) or without surgery (39.07 ± 15.76) is better than that of radical mastectomy (33.84 ± 12.99) or patients with modified radical mastectomy (38.21 ± 13.87) . Reference [15] showed that the visuospatial function, visual memory, and verbal learning of patients with breast cancer chemotherapy were significantly lower than those of patients with surgery alone. At the same time, studies have shown that radiotherapy and other treatments have a superimposing effect, further aggravating the decline of cognitive function. A study by Huehnchen et al. [16] found that radiotherapy can also cause cognitive impairment in patients, and simultaneous radiotherapy and chemotherapy can cause more severe cognitive impairment. One study [17] assessed cognitive function assessment on 60 patients with early breast cancer before surgery, after surgery, before chemotherapy, and after chemotherapy and found that patients at each stage had cognitive dysfunction, indicating that surgery and chemotherapy may both cause cognitive dysfunction. The abovementioned shows that surgery can add to the psychological and physical trauma of breast cancer patients and that different surgical procedures and postoperative radiotherapy can have an impact on cognitive function. In clinical practice, medical staff must pay special attention to patients undergoing radical mastectomy and radiotherapy and, through effective communication and information support, instruct patients to face their illness correctly and avoid the psychological pressure of negative thoughts on patients, improve patients' cognitive function and the quality of life.

## 5. Summary

So far, no drugs are clear and effective for the recovery of cognitive function after chemotherapy. And because of the side effects of neurostimulant drugs, the current research focuses more on cognitive behavioral psychotherapy and other new therapies such as traditional Chinese medicine. Cognitive behavior therapy uses cognitive and behavioral methods to change patients' inappropriate cognition and correct patients' unhealthy behaviors [18]. Chen Xiaomin [19] showed that computer virtual rehabilitation training can improve CRCI, by simulating real game scenes with high interaction with patients, providing personalized treatment plans for different patients to help them improve their cognitive functions. This is consistent with the view of Chai Lijun [20]. Studies have shown that traditional Chinese medicine intervention, reconciliation of qi and blood, and nourishing heart and acupuncture can effectively alleviate and improve the cognitive dysfunction of breast cancer patients after chemotherapy [21, 22]. The research of Tong Taishan [23] also supported this view and further pointed out that acupuncture therapy is mainly manifested in the recovery of patients' subjective cognition, memory, and visual space ability. In addition, high- and low-frequency conversion music therapy and physical exercise can effectively improve the cognitive function of patients with breast cancer chemotherapy and improve the quality of life of patients [24, 25]. In breast cancer chemotherapy patients, with the increase in the number of chemotherapy and the prolongation of the chemotherapy cycle, the cognitive function of the patients is impaired in varying degrees. Clinical medical staff should communicate with patients more, so that patients have a comprehensive understanding of disease-related knowledge, reduce patients' psychological pressure, increase confidence in overcoming the disease, and ultimately promote patients' physical and mental health and improve their quality of life. In the process of CRCI treatment for breast cancer patients, more attention is paid to nondrug treatment, cognitive behavioral psychotherapy, and psychological care and rehabilitation training of patients are paid attention to. Pay attention to the integration of Chinese and Western medicine, give full play to the unique advantages of our country's traditional Chinese medicine industry in the health industry, and strengthen international cooperation in multi-center national and global cooperative researches.

## Figures and Tables

**Table 1:** General demographic data of breast cancer chemotherapy patients (*n* = 172, %).

Factor	Group	Amount of people (*n*)	Composition ratio (%)
*Age (years)*	Scope	26–68	
	Average value (mean ± SD)	49.38 ± 9.20	

*Marriage*	Unmarried	23	13.37
	Married	149	86.63

*Occupation*	Work in city	92	53.49
	Work in rural or unemployed	80	46.51

*Education*	Elementary school and below	52	30.23
	Junior high school	33	19.19
	High school	65	37.79
	University and above	22	12.79

*Monthly income (yuan)*	<1000	15	8.72
	1000–3000	54	31.40
	3001–5000	87	50.58
	>5000	16	9.30

*Family history of breast cancer*	Yes	40	23.26
	No	132	76.74

*Types of breast cancer pathology*	Carcinoma in situ	20	11.63
	Invasive carcinoma	126	73.25
	Other	26	15.12

*Clinical stage*	I	34	19.76
	II	44	25.58
	III	61	35.47
	IV	33	19.19

*Radiotherapy*	Yes	54	31.40
	No	118	68.60

*Surgery*	Yes	145	84.30
	No	27	15.70

*Surgery type*	Radical mastectomy	56	32.56
	Modified radical mastectomy	56	32.56
	Breast conservation	33	19.18
	No surgery	27	15.70

*Metastasis*	Yes	101	58.72
	No	71	41.28

*Time to receive chemotherapy*	Before operation	55	31.98
	After operation	117	68.02

*Current chemotherapy regimen*	CEF	49	28.49
	CET	49	28.49
	TP	21	12.21
	TCH and others	53	30.81

*Number of chemotherapy sessions (times)*	1–9	44	25.58
	10–18	29	16.86
	19–36	62	36.05
	≥37	37	21.51

**Table 2:** Analysis of T-scores of various dimensions and subtests of MCCB (*n* = 172,%).

Cognitive dimension	Subtest	Scope (scores)	Average value (scores, mean ± SD)	Result
Processing speed	Score	21–72	48.83 ± 10.73	Normal
	Category fluency	29–82	62.50 ± 14.79	Extraordinary
	Trail making test	26–80	52.72 ± 12.48	Normal
	Symbolic coding test	10–61	33.31 ± 13.53	Abnormal

Working memory	Score	11–59	36.84 ± 10.25	Abnormal
	Number sequence test	15–67	44.85 ± 9.95	Normal
	Spatial span test	10–49	31.75 ± 12.02	Abnormal

Speech learning	Verbal memory test	12–65	44.67 ± 10.90	Normal
Visual learning	Visual memory	14–64	42.19 ± 9.38	Abnormal
Reasoning and problem solving	Maze test	29–70	50.06 ± 9.08	Normal
Attention/alertness	Continuous operation test	10–68	37.20 ± 12.50	Abnormal
Social cognition	Emotion management test	20–72	39.54 ± 10.17	Abnormal
MCCB		10–63	36.99 ± 13.06	Abnormal

**Table 3:** Ratio analysis of the current status of cognitive dimensions and subtests in patients with breast cancer chemotherapy (*n* = 172,%).

Subtests/dimensions	Result	Frequency	Percentage (%)	Cumulative percentage (%)
*MCCB*	Abnormal	114	66.28	66.28
	Normal	40	23.26	89.54
	Extraordinary	18	10.46	100.00
	In total	172	100.00	

*Working memory*	Abnormal	126	73.26	73.26
	Normal	44	25.58	98.84
	Extraordinary	2	1.16	100.00
	In total	172	100.00	

*Attention/alertness*	Abnormal	121	70.35	70.35
	Normal	43	25.00	95.35
	Extraordinary	8	4.65	100.00
	In total	172	100.00	

*Social cognition*	Abnormal	112	65.12	65.12
	Normal	55	31.98	97.10
	Extraordinary	5	2.90	100.00
	In total	172	100.00	

*Visual memory*	Abnormal	106	61.63	61.63
	Normal	50	29.07	90.70
	Extraordinary	16	9.30	100.00
	In total	172	100.00	

*Verbal memory*	Abnormal	59	34.30	34.30
	Normal	90	52.33	86.63
	Extraordinary	23	13.37	100.00
	In total	172	100.00	

*Processing speed*	Abnormal	47	27.33	27.33
	Normal	81	47.09	74.42
	Extraordinary	44	25.58	100.00
	In total	172	100.00	

*Reasoning and problem-solving*	Abnormal	40	23.26	23.26
	Normal	86	50.00	73.26
	Extraordinary	46	26.74	100.00
	In total	172	100.00	

*Trail making test*	Abnormal	45	26.16	26.16
	Normal	55	31.98	58.14
	Extraordinary	72	41.86	100.00
	In total	172	100.00	

*Symbolic coding test*	Abnormal	136	79.07	79.07
	Normal	30	17.44	96.51
	Extraordinary	6	3.49	100.00
	In total	172	100.00	

*Category fluency test*	Abnormal	23	13.37	13.37
	Normal	40	23.26	36.63
	Extraordinary	109	63.37	100.00
	In total	172	100.00	

*Number sequence test*	Abnormal	57	33.14	33.14
	Normal	93	54.07	87.21
	Extraordinary	22	12.79	100.00
	In total	172	100.00	

*Spatial span test*	Abnormal	139	80.81	80.81
	Normal	32	18.60	99.41
	Extraordinary	1	0.59	100.00
	In total	172	100.00	

**Table 4:** Comparison of scores of various dimensions of cognitive function in breast cancer patients with different characteristics.

Factor	Case (*n*)	Score (mean ± SD)	*t*/*F*	*p*
*Marital status*				
Unmarried	23	32.09 ± 10.99	−1.946	0.053
Married	149	37.99 ± 13.89		

*Place of residence*				
City	92	39.85 ± 13.59	2.777	0.006
Rural	80	34.16 ± 13.18		

*Educational level*				
Elementary school and below	52	25.50 ± 9.37	73.322	≤0.001
Junior high school	33	29.12 ± 8.95		
High school	65	47.09 ± 7.60		
University and above	22	47.77 ± 12.10		

*Monthly income (yuan)*				
<1000	15	32.47 ± 8.44	9.085	≤0.001
1000–3000	54	30.61 ± 12.27		
3001–5000	87	41.32 ± 13.87		
>5000	16	41.50 ± 11.34		

*Pathological type*				
Carcinoma in situ	20	39.55 ± 16.76	0.334	0.717
Invasive carcinoma	126	36.93 ± 13.52		
Metastatic cancer and others	26	36.73 ± 11.99		

*Clinical stage*				
I	34	40.12 ± 17.61	1.979	0.119
II	44	39.16 ± 13.75		
III	61	36.48 ± 11.29		
IV	33	32.94 ± 12.26		

*Surgical approach*				
Radical mastectomy	56	33.84 ± 12.99	1.785	0.152
Modified radical mastectomy	56	38.21 ± 13.87		
Breast conservation	33	39.67 ± 12.00		
No surgery	27	39.07 ± 15.76		

*Timing of chemotherapy*				
Before surgery	55	33.89 ± 13.14	−2.205	0.029
After surgery	117	38.76 ± 13.68		

*Chemotherapy regimen*				
CEF	49	39.49 ± 14.01	2.945	0.035
CET	49	38.49 ± 12.81		
TP	21	29.48 ± 14.45		
TCH	53	36.96 ± 13.04		

*Chemotherapy times*				
1–9	44	48.16 ± 10.56	23.659	≤0.001
10–18	29	41.10 ± 14.15		
19–36	62	32.23 ± 11.76		
≥37	37	29.46 ± 10.00		

**Table 5:** Assignment for multivariate analysis of factors.

Factors	Assignment
Monthly income	1 = <1000, 2 = 1000–3000, 3 = 3001–5000, 4 = >5000
Education level	1 = elementary school and below, 2 = junior high school, 3 = high school, 4 = university and above
Chemotherapy times	1 = 1–9, 2 = 10–18, 3 = 19–36, 4 = ≥37

**Table 6:** Multiple linear regression analysis of cognitive function in patients with breast cancer chemotherapy (*n* = 172).

Model	B	SE	Beta	*t*	*p*	95.0% CI	
						Lower limit	Upper limit
Constant term	21.764	5.343	0.016	4.073	≤0.001	11.213	32.315
Monthly income	3.486	0.985	0.198	3.541	≤0.001	1.542	5.431
Education level	6.718	0.802	0.513	8.378	≤0.001	5.135	8.301
Chemotherapy times	−3.861	0.708	−0.309	−5.455	≤0.001	−5.259	−2.464

Note: *R*^2^ = 0.599, adjust *R*^2^ = 0.579, *F* = 30.455, *p* < 0.001. B is the regression coefficient, SE is the standard error, and 95% CI is the 95% confidence interval.

## Data Availability

The data can be obtained from the author upon reasonable request.
